The article "The Effective Components, Core Targets, and Key Pathways of Ginseng against Alzheimer's Disease" was retracted in 2023. Reasons: signs of a paper mill; compromised peer review; unreliable results or conclusions.

# The Effective Components, Core Targets, and Key Pathways of Ginseng against Alzheimer's Disease

**DOI:** 10.1155/2023/9935942

**Published:** 2023-01-23

**Authors:** Yabo Wang, Xinxin Liu

**Affiliations:** ^1^Department of Neurology, Huaihe Hospital of Henan University, Kaifeng 475000, China; ^2^Department of Geriatrics, First Affiliated Hospital of Henan University, Kaifeng 475000, China

## Abstract

**Background:**

*Panax ginseng* C. A. Mey (*ginseng*) is a traditional Chinese medicinal herb used for the treatment of nervous system disorders, such as Alzheimer's disease (AD). However, the pharmacological mechanisms of *ginseng* involved in AD have not been systematically investigated. Here, a network pharmacology approach was adopted to explore the effective components, core targets, and key pathways of *ginseng* against AD.

**Methods:**

TCMSP database was used to screen the active ingredients of *ginseng*. Prediction of the targets of ginseng and AD-related genes was performed using online public databases. “Compound-Target,” “Compound-Target-Disease,” “Protein-Protein Interaction (PPI),” “Compound-Target-Pathway,” and “Compound-Target-GO–Pathway” networks were constructed with Cytoscape 3.7.2 software. Gene Ontology (GO) function annotation and Kyoto Encyclopedia of Genes and Genomes (KEGG) pathway enrichment were performed by using the DAVID database.

**Results:**

A total of 22 bioactive compounds were identified from *ginseng*, and 481 targets of *ginseng* and 763 AD-related targets were obtained from public databases. The PPI network screened out 19 hub genes of *ginseng* against AD. According to GO function enrichment, ginseng influenced cell proliferation, death, the nitric oxide biosynthetic process, hypoxia response, and synaptic transmission. Neuroactive ligand-receptor interaction, serotonergic synapse, calcium signaling, cAMP signaling, FoxO signaling, Ras signaling, and PI3K-AKT signaling were among the most key regulatory pathways. The compound-target-GO-route network found EGFR, MAPK1, MAPK14, AKT1, CASP3, and PRKACA as key genes, with PI3K-AKT signaling being the most important pathway for ginseng's anti-AD activity.

**Conclusion:**

*Ginseng* exerts neuroprotective effects in AD patients through multicomponent, multitarget, and multipathway modes, providing novel insight into the pharmacological and experimental research on *ginseng* against AD.

## 1. Introduction

Alzheimer's disease (AD) is a chronic neurodegenerative disease and a primary cause of dementia in the aging population worldwide [1]. AD is characterized by a progressive memory deficit, cognitive disorder, loss of acquired learning capacity, compromised daily activity ability, and psychiatric symptoms [2]. The senile plaque formed by aggregation of extracellular *β*-amyloid (A*β*) protein and neurofibrillary tangles triggered by hyperphosphorylation of intracellular tau protein is the typical pathogenesis of AD [3]. Additionally, neuron death, oxidative stress, neurotransmitter dysregulation, and neuroinflammation are also associated with the occurrence and development of AD [4]. As reported, two-thirds of the 50 million cases of dementia worldwide are AD, and the number of dementia cases is expected to reach 152 million by 2050 [5]. In China, it is estimated that there will be 2.35 times more people with AD in 2050 than in 2015, placing a heavy burden on social healthcare costs and families [6]. As FDA-approved anti-AD drugs in clinical practice, acetylcholinesterase inhibitors (AChEIs) and N-methyl-D-aspartic acid (NMDA) receptor antagonists only provide partial symptomatic improvement [7]. Despite the recent approval of aducanumab as the first putative disease-modifying therapy (DMT) for AD, considerable controversy remains over the use of the drug [8]. In view of the complicated pathological mechanisms, multitarget regimens may be a better choice than traditional single-target drugs.

Traditional Chinese medicine (TCM) has evolved and been passed down for thousands of years, forming its theoretical foundation and herb-use features. In TCM, two or more herbs are frequently used for synergism and toxicity reduction. For hundreds of years, TCM, particularly herbal therapy, has been utilized as a supplementary and alternative therapeutic strategy to treat neurodegenerative disorders [9]. *Panax ginseng* C. A. Mey (*ginseng*), a common Chinese herbal medicine, exerts neuroprotective effects against pathological cascades in AD, such as A*β* formation, neuroinflammation, oxidative stress, and mitochondrial dysfunction [10, 11]. As the main active components of *ginseng*, ginsenosides feature antitumor, anti-inflammatory, antioxidant, and antiapoptotic effects [12]. Ginseng protein is one of the active components of ginseng with anti-AD effects in vivo and in vitro [13, 14], and the mechanism of action is associated with the activation of the cyclic adenosine monophosphate/cyclic phosphoadenosine effector element-binding protein (cAMP/CREB) signaling pathway. Brain-derived neurotrophic factor (BDNF) is a CREB downstream effector that binds to tyrosine-protein kinase receptor B (TrkB), causing an increase in TrkB autophosphorylation, which consequently facilitates neuronal growth, survival, and differentiation [15, 16] and protects against neuronal damage elicited by *β*-amyloid (A*β*) [17]. The BDNF/TrkB signaling pathway is closely related to cognitive function, and inactivation of this pathway may lead to abnormal cognitive function [18]. Also, BDNF expression is closely associated with gut microbes, and disturbances in the gut flora reduce BDNF levels in the cerebral cortex and hippocampus, thereby leading to dysfunction of the central nervous system, behavioral abnormalities, cognitive impairment, or even AD [19].

Nevertheless, *ginseng* or ginsenosides have been frequently investigated in single-target studies. For instance, *ginseng* improved the memory ability and decreased the level of A*β*_1–42_ and p-tau in AD rats by activating PI3K/AKT signaling pathway [20], ginsenoside Rg1 lowered A*β* contents via suppressing CDΚ5-mediated PPAR*γ* phosphorylation in a neuron model of AD [21], and ginsenoside Rg2 protected against A*β*_25–35_-induced apoptosis in AD by the enhancement of PI3K/Akt signaling pathway [22]. However, single-target research is insufficient to fully understand the entire medicinal effects and mechanism of action of ginseng for AD therapy. As a result, proper multitarget research is required to thoroughly explore the mechanisms of ginseng in AD.

Network pharmacology is an integrated approach based on pharmacology, network biology, systems biology, bioinformatics, and computational science [23]. It is widely applied to reveal the action mechanism of TCM through establishing a “drug-component-target-disease” interaction network [24]. Accordingly, the present study employs a new network pharmacology approach to investigate the interaction between drug and target by searching databases of genes, proteins, illnesses, and medications, as well as real experimental data, to establish a relationship network between “drug-gene-target-disease.” It is envisaged that medications will be able to rebalance the biological network to investigate the influence of ginseng against AD. Furthermore, the integrity and systematic character of pharmacological research strategy of the TCM network, in accordance with the principles of disease diagnosis and treatment, is also a feature of the synergistic action of multicomponents, multiapproaches, and multitargets in TCM and its prescriptions.

## 2. Materials and Methods

### 2.1. Screening of Active Ingredients in *Ginseng*

Traditional Chinese Medicine Systems Pharmacology (TCMSP) database (https://old.tcmsp-e.com/tcmsp.php) [25] was used to select the chemical compounds with the keywords of “Panax *Ginseng* C. A. Mey.” The absorption, distribution, metabolism, and excretion (ADME) model were used to predict the pharmacokinetic properties of natural compounds. The bioactive components were screened from *ginseng* as per the criteria of oral bioavailability (OB) ≥30% and drug-likeness (DL) ≥0.18.

### 2.2. Collecting Potential Targets Related to Bioactive Ingredients of *Ginseng*

The relevant targets of the active components of *ginseng* were obtained by using the TCMSP database. PharmMapper (https://www.lilab-ecust.cn/pharmmapper/submitfile.html) [26] and TargetNet [27] were also employed to acquire compound-related targets. Firstly, PubChem (https://pubchem.ncbi.nlm.nih.gov/) and TCMSP were used to collect the canonical smiles and mol2 structure files, respectively. The protein structure in mol2 format was uploaded to PharmMapper with the limitations of “Homo sapiens” and “normal fit score >0.6.” Then, canonical smiles were imported into TargetNet with limitations of “Homo sapiens” and “probability >0.8.” UniProt database (https://www.uniprot.org/) [28] was adopted to obtain the corresponding gene symbols with species limited to “Homo sapiens.” After ruling out the duplicates, all putative targets of *ginseng* were obtained.

### 2.3. Identification of Candidate Targets for AD

The AD-related genes were retrieved from 5 public databases, including GeneCards (https://www.genecards.org/) [29], DisGeNET (https://www.disgenet.org/) [30], AlzPlatform (https://www.cbligand.org/AD/) [24], DrugBank (https://www.drugbank.ca/) [31], and Therapeutic Target Database (TTD) (https://db.idrblab.net/ttd/) [32], with the search term of “Alzheimer's disease.” All targets were standardized to the UniProtKB form. The final AD target genes were acquired after removing the repetitive items.

### 2.4. Network Establishment

#### 2.4.1. “Compound-Target (C-T)” Network of *Ginseng*

The active components and corresponding targets of *ginseng* were introduced into Cytoscape 3.7.2 to construct this network.

#### 2.4.2. “Compound-Target-Disease (C-T-D)” Network

An online Venn diagram tool (https://bioinformatics.psb.ugent.be/webtools/Venn/) was used to obtain the intersection of *ginseng*- and AD-related genes. Then, the active ingredients, diseases, and overlapping targets were entered into Cytoscape 3.7.2 to establish this network.

#### 2.4.3. “Protein-Protein Interaction (PPI)” Network

Although PPI networks are less closely associated with mRNA expressions, the goal of the present study after differential analysis was to identify hub genes using the PPI network, which had no implications for the results. The intersection targets were imported into the STRING database (https://string-db.org/) [33] to analyze the interaction between proteins with “Homo sapiens” and “minimum required interaction score >0.7.” The TSV files were downloaded from the STRING database and imported into Cytoscape 3.7.2 software for PPI analysis and visualization. The topological importance of the nodes in the network was evaluated with three important topological parameters, namely, betweenness centrality (BC), closeness centrality (CC), and degree centrality (DC). The two rounds of screening for hub genes were performed based on threshold values of BC, CC, and DC ≥median values.

#### 2.4.4. “Compound-Target-Pathway (C-T-P)” Network

The pathway annotation of overlapping genes was conducted using KEGG pathway enrichment analysis. The active components, target proteins, and pathway information were introduced into Cytoscape 3.7.2 to establish the CTP network.

#### 2.4.5. “Compound-Target-GO-Pathway (C-T-G-P)” Network

The 17 key genes from the PPI network, corresponding active components, top 20 GO terms, and top 25 pathways were imported into Cytoscape software to construct the C-T-G-P integrative network.

### 2.5. GO Function and KEGG Pathway Enrichment Analysis

Online bioinformatics tool DAVID (https://david.ncifcrf.gov/) [34] was utilized for GO function and KEGG pathway enrichment analysis of drug-disease common targets. When *P* < 0.05, the enriched terms were considered significantly significant. The top 20 relevant biological processes and top 30 KEGG pathways were displayed as bubble charts by using online tool bioinformatics (https://www.bioinformatics.com.cn/). The KEGG mapper (https://www.kegg.jp/kegg/mapper/) was employed to analyze the upstream and downstream genes of crucial signaling pathways.

## 3. Results

### 3.1. Screening of Bioactive Components from *Ginseng*

A total of 190 chemical ingredients were identified in *ginseng*. After ADME screening with OB ≥30% and DL ≥0.18, 22 active components of *ginseng* were finally obtained (Figure 1 and Table 1).

### 3.2. Collection of Potential Targets for Bioactive Ingredients of *Ginseng*

TCMSP, PharmMapper, and TargetNet were used to predict the potential targets of 22 bioactive components. There were 117 targets from TCMSP, 256 targets from PharmMapper (norm fit >0.6), and 206 targets from TargetNet (probability >0.8). After ruling out the duplicate targets, the remaining 481 targets were identified as the candidate targets of *ginseng*. The detailed information is shown in Supplemental Table S1. By using Cytoscape 3.7.2, a “Compound-Target” network was established (Figure 2). In this network, there were 503 nodes and 2793 edges. The ginseng active components were represented by yellow arrow nodes and the targets by green diamond nodes, illustrating the interaction between chemical compounds and probable targets. The top ten constituents are presented below in order of degree: MOL005320 (arachidonate, degree = 208); MOL005318 (dianthramine, degree = 199); MOL002879 (Diop, degree = 171); MOL005344 (dinsenoside rh2, degree = 168); MOL004492 (chrysanthemaxanthin, degree = 161); MOL000422 (kaempferol, degree = 160); MOL005360 (malkangunin, degree = 159); MOL005376 (panaxadiol, degree = 141); MOL000358 (beta-sitosterol, degree = 133); and MOL000449 (stigmasterol, degree = 127).

### 3.3. Interactional Network Analysis of Active Compound Targets and AD-Targets

GeneCards, DisGeNET, AlzPlatform, DrugBank, and TTD databases were employed to predict targets related to AD. There were 363 targets from GeneCards (relevance score ≥20), 154 targets from DisGeNET (Score_gda >0.2), 320 targets from AlzPlatform, 89 targets from DrugBank, and 131 targets from TTD. After excluding duplicates, 763 targets were found to be linked to AD, as shown in Supplementary Table S2. The Venn diagram showed that a total of 177 targets may be implicated in ginseng therapy for AD (Figure 3(a) and Supplemental Table S3). Through Cytoscape 3.7.2, a “Compound-Target-Disease” network was constructed (Figure 3(b)), among which there were 201 nodes and 1318 edges. These data suggested that *ginseng* might affect AD through these bioactive compounds to regulate multiple targets.

### 3.4. PPI Network Construction

The 177 common targets were inputted into the STRING database and Cytoscape 3.7.2 software to establish a PPI network of compound targets and AD targets. This network consisted of 166 nodes and 845 edges (Figure 4(a)), among which nodes and edges represent interacting proteins and interactions, respectively. The topological properties of this PPI network were analyzed based on three major network parameters of “BC,” “CC,” and “DC.” The targets with BC, CC, and DC exceeding median values were identified as hub genes to establish the core network of *ginseng* against AD. The cutoff values of the first screening were DC ≥ 9, CC ≥ 0.399, and BC ≥ 0.0024, with the results of 53 nodes and 322 edges (Figure 4(b)). Subsequently, the 53 targets were further processed with threshold values as degree ≥11, CC ≥ 0.5, and BC ≥ 0.0084, and 19 nodes and 86 edges were finally obtained (Figure 4(c)). The node size and color are proportionate to the degree. The bigger and darker the node, the more significant it is in the hub network. MAPK1, TNF, EGFR, AKT1, and IL2 may account for the important therapeutic benefits of ginseng against AD as the target genes with the highest degree values.

### 3.5. Biological Functions and Pathways Enrichment

To further illustrate the action mechanism of *ginseng* on AD, the 177 common targets were imported into the DAVID database for GO function and KEGG pathway enrichment. When *P* ≤ 0.05, the GO terms and KEGG pathways were considered significantly enriched. The results showed a variety of GO enrichment terms, including 441 biological processes (BP), 54 cell components (CC), and 103 molecular functions (MF) items. The GO information is displayed in detail in Supplemental Table S4. The top 15 significantly enriched GO terms in BP, CC, and MF were plotted and visualized into a bar graph (Figure 5(a)), indicating that *ginseng* might regulate cell proliferation, apoptosis, nitric oxide biosynthetic process, response to hypoxia, and synaptic transmission via enzyme binding, protein tyrosine kinase activity, heme binding, and oxygen binding in the plasma membrane, membrane raft, dendrite, extracellular space, and cytosol to exert its anti-AD effects. The top 20 biological processes were used to draw a bubble chart (Figure 5(b)). In addition, a total of 113 related pathways were identified (Supplemental Table S5). The most significantly enriched 30 pathways involved in *ginseng* against AD are shown in Figure 5(c), including neuroactive ligand-receptor interaction, serotonergic synapse, calcium signaling pathway, cAMP signaling pathway, FoxO signaling pathway, Ras signaling pathway, PI3K-AKT signaling pathway, Rap1 signaling pathway, TNF signaling pathway, HIF-1 signaling pathway, and cGMP-PKG signaling pathway. The important genes were mainly enriched in the PI3K-AKT signaling pathway (Figure 6).

### 3.6. Compound-Target-Pathway Network Analysis

A compound-target-pathway network was built with the bioactive components, top 25 signal pathways (Supplemental Table S5), and corresponding target genes. In this network, there were 174 nodes and 1225 edges (Figure 7). The yellow arrows, green diamonds, and orange hexagons represent active ingredients, targets, and regulatory pathways, respectively. According to the degree number, 11 components including MOL005318 (dianthramine), MOL002879 (Diop), MOL000422 (kaempferol), MOL000358 (beta-sitosterol), MOL005320 (arachidonate), MOL005344 (ginsenoside rh2), MOL000449 (stigmasterol), MOL004492 (chrysanthemaxanthin), MOL005384 (suchilactone), and MOL005321 (frutinone A) were considered of great significance. Targets serve as links between chemicals and pathways. MAPK1, MAPK14, EGFR, PRKACA, AKT1, AR, ESR1, CASP3, BRAF, and NOS3 were the top 20 targets in the compound-target-pathway network. The key pathways implicated in *ginseng* against AD were hsa04080 (neuroactive ligand-receptor interaction), hsa04020 (calcium signaling pathway), hsa04151 (PI3K-Akt signaling pathway), hsa04726 (serotonergic synapse), hsa04024 (cAMP signaling pathway), hsa04014 (Ras signaling pathway), hsa04015 (Rap1 signaling pathway), and hsa04068 (FoxO signaling pathway). These data suggested the multiple components, multiple targets, and multiple pathways of *ginseng* in preventing AD.

### 3.7. Compound-Target-GO-Pathway Network Analysis

The top 25 KEGG pathways, top 20 GO terms, 17 common targets, and active components were input into Cytoscape software to construct the “C-T-G-P” integrative network, and 82 nodes and 308 edges were observed in this network (Figure 8). MOL000422 (kaempferol), MOL005318 (dianthramine), MOL005344 (ginsenoside rh2), MOL004492 (chrysanthemaxanthin), MOL005320 (arachidonate), MOL000358 (beta-sitosterol), MOL000449 (stigmasterol), and MOL002879 (Diop) were identified as the key compounds. EGFR, MAPK1, MAPK14, AKT1, CASP3, and PRKACA were identified as kernel targets. GO:0005886 (plasma membrane) and GO:0007165 (signal transduction) were the most important GO terms. hsa04151 (PI3K-Akt signaling pathway) was the most crucial pathway.

## 4. Discussion

AD is a complicated and progressive neurodegenerative disorder with multiple pathophysiological mechanisms [35]. *Ginseng* is a TCM herb with pharmacological activities and is considered beneficial for neurological damage and related diseases, including AD [1]. A thorough network pharmacology analysis was performed in the current study to investigate the underlying processes and therapeutic targets of *ginseng* in AD. The findings identified 22 chemical components, 19 key targets, 441 biological processes, and 113 related signal pathways for *ginseng* in the treatment of AD. Compound-target-pathway network identified MAPK1, MAPK14, EGFR, PRKACA, AKT1, CASP3, and NOS3 as core targets of *ginseng* against AD.

Twenty two chemical components of *ginseng* were identified as per the criteria of OB ≥30% and DL ≥0.18. In the present study, a compound-target network of *ginseng* was established. This network showed that each component could yield complications on multiple targets. For example, Arachidonate, dianthramine, Diop, Ginsenoside rh2, Chrysanthemaxanthin, and Kaempferol, respectively, acted on 208, 199, 171, 168, 161, and 160 targets. Also, most active components act on the same targets. These results indicated the multicomponent and multitarget action mode of *ginseng*. Some of these compounds have been documented to exert a suppressive effect on central nervous system diseases, including AD. Moreover, exposure of AD flies to kaempferol resulted in the loss of climbing and memory ability, lowered oxidative stress, and inhibited acetylcholinesterase activity [36]. A recent report found that the administration of *β*-sitosterol in amyloid protein precursor/presenilin 1 (APP/PS1) mice could decrease A*β* deposition and mitigate cognitive impairment [37]. Ginsenoside Rh2 exhibited neuroprotective effects against scopolamine-induced memory deficits in mice possibly through regulating cholinergic transmission, oxidative stress, and the ERK-CREB-BDNF signaling pathway [38]. Stigmasterol could protect against oxidative stress-induced neuronal cell death via the sirtuin family, suggesting the potential of stigmasterol to alleviate neurodegeneration [39]. Panaxadiol was revealed to reduce synaptic damage in AD via inactivating the Fyn/GluN2B/CaMKII*α* signaling pathway [40]. Ginsenoside Rg5 alleviated cognitive deficits and A*β* deposition in streptozotocin (STZ)-induced rats through repressing neuroinflammatory responses [41]. Inflammation [42], oxidative stress [43], and apoptosis [44] are considered vital risk factors for the onset and progression of AD. Hence, they might play a neuroprotective role in AD by modulating inflammation, oxidative stress, and apoptosis.

A PPI network of *ginseng* against AD was constructed, with the results of 166 nodes and 845 edges. Based on the topological parameters, 19 hub genes (MAPK1, TNF, EGFR, AKT1, IL2, MAPK14, NOS3, IGF1, CASP3, FYN, PTGS2, APP, IL1B, ALB, HSP90AA1, JAK2, CXCR2, PRKACA, and CHRM2) were obtained. Activation of the TNF pathway mediated by miR-206 promotes the production and release of inflammatory mediators such as TNF-*α*, IL-8, and IL-6 by driving NF-*κ*B into the nucleus, thereby participating in inflammatory and immune processes [45]. The high presence of TNF inflammatory cytokines in the tumor microenvironment promotes tumor growth, disrupts cell proliferation and death, and impairs the innate immune response to cancer cells [46]. These studies all demonstrate the reliability of the current experimental results. Numerous studies have revealed that TNF-*α* activates JAK/STAT signal pathway via the protein-gp130 on the cell membrane surface and facilitates the control of degenerative alterations in the central nervous system [47].

Based on the data from GO analysis, *ginseng* was implicated in AD progression possibly via affecting cell proliferation, apoptosis, nitric oxide biosynthetic process, response to hypoxia, and synaptic transmission. The KEGG enrichment analysis found that the main mechanisms of *ginseng* against AD were neuroactive ligand-receptor interaction, serotonergic synapse, calcium signaling pathway, cAMP signaling pathway, FoxO signaling pathway, Ras signaling pathway, PI3K-AKT signaling pathway, and Rap1 signaling pathway. The neuroactive ligand-receptor interaction signaling pathway is associated with neurological diseases, such as Parkinson's disease (PD) [48] and glioblastoma [49]. Disruption of calcium signaling may trigger synaptic deficits and induce the accumulation of A*β* plaques and neurofibrillary tangles in AD [50]. cAMP/PKA signaling pathway contributed to neuronal apoptosis and A*β* accumulation in a mixed model in Type 2 diabetes (T2D) and AD through regulating IDE expression [51]. FoxO proteins, a family of transcription factors with 4 members (FOXO1, FOXO3a, FOXO4, and FOXO6), protect multiple cells in the brain by controlling autophagy and apoptosis, highlighting FoxO as a biomarker and potential target for AD treatment [52]. Inhibition of Ras-MAPK signaling suppressed the hyperphosphorylation of tau and amyloid precursor protein (APP) as well as neuronal cell cycle entry in AD [53]. Thereby, *ginseng* might slow down AD progression via regulating oxidative stress, apoptosis, and synaptic transmission through these related signaling pathways.

To elucidate the key targets of *ginseng* against AD in the related pathways, a “compound-target-GO-pathway” network was also built up, and 6 core targets including EGFR, MAPK1, MAPK14, AKT1, CASP3, and PRKACA were obtained. MAPK1 and MAPK14, members of the MAPK family, regulate various cellular activities, such as oxidative stress, inflammatory reaction, immune response, apoptosis, proliferation, and survival [54]. p38 MAPK can control tau phosphorylation, neurotoxicity, neuroinflammation, and synaptic dysfunction associated with AD [55]. EGFR, expressed in both central and peripheral nervous systems, possesses specific important neurotrophic functions, particularly in the central nervous system [56]. Inhibition of EGFR decreases reactive astrocytes, induces autophagy, weakens A*β* toxicity and neuroinflammation, and regenerates axonal degradation in AD [57]. PKA, encoded by PRKACA, is found to exert a neuroprotective effect in a cell culture model of AD [49]. Activation of the PKA/SIRT1 signaling pathway by photobiomodulation therapy decreases A*β* levels in AD [58]. Caspase-3 is a key mediator of neuronal programmed cell death in many chronic neurodegenerative diseases [59] and is involved in the regulation of multi-neuro-degenerative disorders, including AD [60]. Moreover, PI3K-AKT signaling was identified as the most important pathway involved in *ginseng* against AD. PI3K/AKT signaling pathway is a critical regulator for various signal transduction and biological processes such as cell proliferation, apoptosis, and metabolism. PI3K/AKT signal pathway is found to be involved in the formation of two special pathological structures in AD [61]. Various downstream targets of this pathway are closely related to the occurrence and development of AD [62, 63]. PI3K-Akt signal pathway activates PI3K by promoting Akt phosphocreatine and regulates cell proliferation to facilitate tumor growth [64]. In addition, aerobic glycolysis, as a unique metabolic mode of tumor, provides substantial carbon sources for tumor tissue for proliferation and inhibits the aerobic oxidation pathway to avoid the production of oxygen radicals and apoptosis, in which PI3K/Akt signaling pathway plays an important role [65].

Natural products, such as flavonoids, alkaloids, phenylpropanoids, and glycosides, are widely used for the prevention and treatment of AD based on the PI3K/AKT pathway [66–68]. This study demonstrates the features of active components, multiple targets, and different routes in ginseng for Alzheimer's disease. However, more extensive experimental validation is required prior to the clinical promotion of *ginseng* in the treatment of Alzheimer's disease.

Although this study provides some ideas for *ginseng* against Alzheimer's disease, it has some limitations. (1) We only used the TCMSP database. Although the drugs included in this database are relatively comprehensive, it has not been updated for a long time, and there may be some new discoveries or newly identified active ingredients are not included. We will synthesize multiple databases such as TCMID, ETCM, and YaTCM to complement drug targets. We will also supplement the literature. (2) Only the disease database was included in this study. Although these are the disease targets of Alzheimer's disease, they still lack specificity relative to the differential genes compared with healthy people. We will perform a variance analysis to enrich the content. (3) We only carried out the bond energy of molecular docking for the compound, lacking specific molecular docking, and the weight is not great although it has a certain impact.

## 5. Conclusion

A network pharmacology approach was utilized to elucidate the target genes and underlying molecular mechanisms of *ginseng* against AD. Kaempferol, dianthramine, ginsenoside rh2, chrysanthemaxanthin, arachidonate, beta-sitosterol, stigmasterol, and Diop are considered the main active compounds of *ginseng*. Ginseng may act as a regulator via the PI3K-AKT signaling pathway. The primary targets identified were EGFR, MAPK1, MAPK14, AKT1, CASP3, and PRKACA, and ginseng and its constituents may have therapeutic promise for Alzheimer's disease.

## Figures and Tables

**Figure 1:** Flowchart of the network pharmacology analysis for *ginseng* against AD.

**Figure 2:** Compound-target network of *ginseng*. Yellow arrows represent 22 active components and green diamonds represent 503 putative targets. The larger the size of compound nodes, the more of the number of degrees.

**Figure 3:** (a) Venn diagram showing the overlapping genes of *ginseng*-targets and AD-targets. (b) Compound-target-disease network. The purple octagon stands for *ginseng*, the yellow arrows stands for the compounds of *ginseng,* the green diamond stands for targets, and the orange circle stands for AD.

**Figure 4:** Identification of core targets of *ginseng* against AD. (a) The interactive PPI network of *ginseng* putative targets and AD-related targets. (b) PPI network of important targets extracted from A. (c) PPI network of core targets of *ginseng* against AD. DC, degree centrality; CC, closeness centrality; BC, betweenness centrality.

**Figure 5:** GO function annotation and KEGG pathway enrichment. (a) GO second class enrichment analysis of 177 common targets for against AD. (b) Bubble plot of top 20 enriched biological processes (BP). (c) Bubble plot of top 30 enriched signaling pathways.

**Figure 6:** The core genes of *ginseng* against AD are mainly distributed in PI3K-AKT signaling pathway. The red nodes are representative for the intersection genes.

**Figure 7:** Compound-target-pathway network of *ginseng* against AD. The yellow arrow nodes represent the compounds, the green diamond nodes represent the targets, and the orange hexagon nodes represent the regulatory pathways.

**Figure 8:** Compound-target-GO-pathway network of *ginseng* against AD. The yellow arrow nodes represent the compounds, the green diamond nodes represent the targets, the blue circles represent the GO terms, and the orange hexagon nodes represent the regulatory pathways.

**Table 1:** Potential active components of *ginseng*.

Mol ID	Molecule name	MW	OB (%)	DL
MOL002879	Diop	390.62	43.59	0.39
MOL000449	Stigmasterol	412.77	43.83	0.76
MOL000358	Beta-sitosterol	414.79	36.91	0.75
MOL003648	Inermin	284.28	65.83	0.54
MOL000422	Kaempferol	286.25	41.88	0.24
MOL004492	Chrysanthemaxanthin	584.96	38.72	0.58
MOL005308	Aposiopolamine	271.34	66.65	0.22
MOL005314	Celabenzine	379.55	101.88	0.49
MOL005317	Deoxyharringtonine	515.66	39.27	0.81
MOL005318	Dianthramine	289.26	40.45	0.2
MOL005320	Arachidonate	304.52	45.57	0.2
MOL005321	Frutinone A	264.24	65.9	0.34
MOL005344	Ginsenoside rh2	622.98	36.32	0.56
MOL005348	Ginsenoside-Rh4_qt	458.8	31.11	0.78
MOL005356	Girinimbin	263.36	61.22	0.31
MOL005357	Gomisin B	514.62	31.99	0.83
MOL005360	Malkangunin	432.56	57.71	0.63
MOL005376	Panaxadiol	460.82	33.09	0.79
MOL005384	Suchilactone	368.41	57.52	0.56
MOL005399	Alexandrin_qt	414.79	36.91	0.75
MOL005401	Ginsenoside Rg5_qt	442.8	39.56	0.79
MOL000787	Fumarine	353.4	59.26	0.83

## Data Availability

The datasets used during the present study are available from the corresponding author upon reasonable request.

## Supplementary Materials

Supplementary Materials Table S1: putative targets for bioactive compounds from *ginseng*. Table S2: AD-related target genes. Table S3: the *ginseng*-AD common targets. Table S4: the GO function enrichment analysis. Table S5: the KEGG pathway enrichment analysis.
